The article "The Application of Magnetic Resonance Imaging in Skeletal Age Assessment" was retracted in 2023. Reasons: signs of a paper mill; suspected computer-generated content; unreliable results or conclusions; lack of ethics approval or compliance.

# The Application of Magnetic Resonance Imaging in Skeletal Age Assessment

**DOI:** 10.1155/2022/9607237

**Published:** 2022-02-21

**Authors:** Khalaf Alshamrani

**Affiliations:** Radiological Sciences Department, College of Applied Medical Science, Najran University, Najran, Saudi Arabia

## Abstract

**Method:**

The study includes 80 patients identified from an endocrine clinic, two males and two females from each of 5 age groups (<5, 5 to 7, 8 to 10, 11 to 13, and 14 to 16 years). Skeletal age as determined from an open MRI scanner and radiographs performed on the same day was compared for each child. Two observers assess the skeletal age from radiographs and MRI images independently. After a period of at least three weeks, observers determined the skeletal age of all patients independently. All of the images were in different and random orders, on both of the assessment occasions. The agreement was assessed using the interclass correlation coefficient and Bland Altman plots. *Problem Statement*. The recurrent use of left-hand radiography in children with chronic conditions might result in the patient being exposed to the same image several times throughout the course of their lives. Use of radiation-free methods such as magnetic resonance imaging (MRI) may be able to assist in reducing the risks associated with radiation exposure, if done properly.

**Results:**

Patients' age ranged from 3 to 16 years, in which the mean of the chronological age was 9.3 years (±2.9) and 9.8 years (±2.7) in girls and boys, respectively. The interrater agreement for skeletal age determination was 0.984 for radiographs and 0.976 for MRI scans. Using the G&P technique, for Observer 1, intraobserver agreement for radiographs and DXA was 0.993 and 0.983, respectively, and 0.995 and 0.994, respectively, for Observer 2. Plotting the rater readings against the line of equality shows no significant differences between readings acquired from radiographs and MRI scans.

**Conclusion:**

For the study contribution, it is possible to employ open compact MRI to determine the skeletal age of a person. Our results showed that left-hand MRI scans were of better quality than the radiographs.

## 1. Introduction

There are different methods currently in practice to assess skeletal maturation. One of the commonest and fastest methods is the assessment of skeletal age from left-hand radiographs [1, 2]. The method is based on the fact that the ossification of the bones appears and fuses at different chronological ages; these then can be captured at different times to reflect the skeletal age [3]. Furthermore, different techniques and atlas have been developed to reflect the skeletal age of healthy children during their childhood. The Greulich & Pyle (G&P) atlas is one of the most commonly used methods when it comes to determining skeletal age from left-hand radiographs [4]. The method required that a radiograph is compared to different standard plats illustrated by the G&P atlas in which the most resemblance plats is chosen then a skeletal age is given to the patient.

The G&P method has been criticised for being outdated in which the applicability of the method to the current population is questionable [5]. Despite this, several studies have shown that ethnicity of the population, as well as socioeconomic characteristics, might contribute to the method's inapplicability [5–10], for example). Because of this, an update to the G&P approach or the adoption of a local standard might help to resolve these problems. Magnetic resonance imaging (MRI) is advantageous in situations when patients are more susceptible to ionizing radiation, such as those involving cancer patients [11].

Theoretically, this can contribute to a better visualization of the bone and cartilages, which is mainly evaluated in skeletal age assessment. Several studies have compared the use of MRI to conventional X-ray imaging for the purpose of skeletal age assessment [12–14]. Overall, the results are encouraging which can offer an alternative method for skeletal age determination. However, the majority of these studies used enclosed scanners that have a higher magnetic field between 1 and 1.5 T. Nevertheless, the open MRI scanners, which have an additional advantage of less discomfort and claustrophobic for children, could be particularly well suited for skeletal age assessment. A study by Terada et al., which used an open 0.3 T MRI scanner, suggested that skeletal age can be determined using an open MRI [15]. However, the study did not compare the results to the gold standard which is the hand-wrist radiograph, and the study results can only be applied to the TW2 method.

Children with chronic diseases are often subjected to repeated left-hand radiography throughout their youth, which might result in the patient being exposed to the same picture several times over the course of their life. It is possible that using radiation-free techniques, such as magnetic resonance imaging (MRI), may help to limit the dangers associated with radiation exposure [16]. Aside from that, it is feasible to complete the process of defining a local bone maturation standard without exposing otherwise healthy children to hazardous amounts of radioactivity [17–20].

## 2. Materials and Methods

### 2.1. Study Design

The study recruited 80 patients divided into 5 age groups in which patients' age ranged from 5 to 16 years. Children referred for different clinical indications to the diagnostic radiological department at [anonymised] to have left-hand radiographs were included. Only patients with their parents who provided full consent were recruited to the study.

After obtaining informed consent, the left-hand radiograph is taken by including at least 1 inch of the distal part of the forearm as well as hand and wrist on the radiation field. According to the patient age, the exposure factors were adjusted which generally ranged from 40 to 42 kV for the tube voltage, 1.7 mAs, FFD 1.05 m. Once the radiographs are taken, patients would immediately have the left-hand MRI scan. The coronal sequences were performed as follows: the left hand and wrist are at the side of the patient, and the middle finger is on the same axis as the forearm.

To ensure that patient corresponding images are not indefinable, all of the radiographs and MRI images were anonymised. Then, two observers assess the skeletal age from radiographs and MRI images independently. After a period of at least three weeks, observers determined the skeletal age of all patients independently. All of the images were in different and random orders, on both of the assessment occasions.

### 2.2. Image Quality Assessment

The adequacy and quality of hand positioning were rated using the Hawley et al. method [21]. The method rates the adequacy in terms of the following:

- Including all of the anatomical area within the hand on the radiation field
- Position of the thumb
- Position of the fingers

These are rated on a system of a 3-point scale (1 = poor, 2 = moderate, and 3 = good) which can generate a possible total score of 9. The image that scored 4 or less is deemed to be of poor hand positioning. Images that scored between 5 and 7 are of adequate positioning while a score between 8 and 9 is deemed to be of good positioning. In terms of image quality, a method described by Cockill et al. was used to determine the overall image quality [22].

### 2.3. Statistical Analysis

The interclass correlation coefficient (ICC) was used to evaluate the agreement between modalities using readings for radiographs and for MRI images from the two observers. To further illustrate the correlation between the radiograph and MRI images, Bland Altman plots were performed [23–25]. The statistical difference between radiographs and MRI images regarding the image quality was evaluated by a paired *t* test.

## 3. Results

Patients' age ranged from 3 to 16 years, in which the mean of the chronological age was 9.3 years (±2.9) and 9.8 years (±2.7) in girls and boys, respectively. The agreement between observers and for each observer using the intra-inter-observer reliability test is presented in Table 1. The mean of skeletal age per age group in males and females using radiographs and MRI images is shown in Table 2.

A significant statistical difference (*p* < 0.001) between left-hand MRI and radiographs was noticed in terms of the quality and adequacy of positioning (Table 3). Regarding hand positioning, around 78% (63) of the hand radiographs were of good positioning compared to 61% (49) of the MRI scans. Nevertheless, only 8% [7] of the hand MRI scans had a poor positioning rating. The score of all of the hand positioning when radiographs were rated had a mean of 8.05 (±0.78) compared to 7.02 (±1.02) for MRI images. Regarding the quality, rating radiographs showed an overall mean of 3.42 (±0.95) compared to 4.11 (±0.48) in MRI images.

Differences between skeletal age assessment from MRI scans and radiographs showed a normal distribution. Differences between the two methods for each observer are illustrated in Figures 1 and 2. The line of equality shows no significant differences between readings acquired from radiographs and MRI scans (Figure 3).

## 4. Discussion

Skeletal age assessment is required for managing children with certain growth disorders and essential in certain cases in which planning for therapeutic interventional procedures is required during childhood. The left-hand radiograph has been commonly used for skeletal age assessment. The G&P method offers a faster and easier approach for the assessment of the skeletal age which increases the popularity of the method among paediatricians [26]. However, patients who required regular skeletal age monitoring are more likely to be exposed to much ionizing radiation during their childhood. To eliminate the risk of exposure to radiation involved in this particular assessment, we aimed to evaluate the possibility of assessing skeletal age using left-hand MRI images.

Firstly, our results showed high inter- and intraobserver agreement between MRI and radiographs. When plotting the mean of the skeletal age acquired from radiographs and MRI against the line of equality, the correlation was high. Our results suggest that the determination of skeletal age using MRI images has no significant difference from those determined from radiographs. Previous studies found that skeletal age from MRI scans and radiographs has reported a high correlation when using an enclosed MRI [27, 28]. Nevertheless, this study showed that open MRI units are able to provide a comparable result to enclosed units with the advantage of being less claustrophobic for children.

The differences between the skeletal age from MRI images and radiographs were in the range of one year; however, certain cases were within the range of 2 years. This is more likely to be due to poor hand positioning during MRI scan, which eventually impacts the image quality. The scanning time could also be the source of the inadequacy of hand positioning in which MRI scanning was on average 1.45 minutes compared to 1 second for a radiograph. This higher time increases the probability of patient movement especially in the case of younger children who are less cooperative. This can lead the child to move his/her hand during the scan which resulted in the exclusion of the ulna and disturbing the image resolution. The visualization of soft tissue and cortical edge was highly rated in MRI images compared to radiographs, which offer an advantage when assessing whether the growth plates fused or not.

Several studies have suggested that, to accurately assess child growth, a regional skeletal maturation atlas representing those children is needed [29–31]. MRI can facilitate the establishment of such a standard without exposing healthy children to ionizing radiation. However, in this study, assessing skeletal age using MRI images took more time than determining skeletal age from radiographs. This is because assessing individual MRI images for each left-hand scan requires more time to view the different maturity markers. In contrast, a radiograph is a single image in which the maturity markers can be assessed easily. Another limitation is the motion artefact within some of the MRI scans. This is mainly due to the difficulty in keeping younger children still during the scan although parental support was there.

## 5. Conclusion

For the study contribution, it is possible to employ open compact MRI to determine the skeletal age of a person. Our results showed that left-hand MRI scans were of better quality than the radiographs.

## Figures and Tables

**Figure 1:** The variation between MRI and radiograph reading for Rater 1 using Bland Altman plot.

**Figure 2:** The variation between MRI and radiograph reading for Rater 2 using Bland Altman plot.

**Figure 3:** The mean of skeletal age for MRI and radiographs when plotted against line of equality.

**Table 1:** The mean skeletal age assessment based on MRI vs. radiographs.

Age group	Skeletal age (years, months)			
	Radiographs		MRI	
	Observer 1	Observer 2	Observer 1	Observer 2
Less than 5 y	4.6 (±0.43)	4.8 (±0.48)	4.7 (±0.53)	4.4 (±0.46)
5 to 7 years	6.3 (±0.52)	6.1 (±0.42)	6.4 (±0.59)	6.5 (±0.63)
8 to 10 years	8.7 (±0.62)	8.5 (±0.58)	8.4 (±0.72)	8.2 (±0.66)
11 to 13 years	12.4 (±0.57)	12.5 (±0.60)	12.2 (±0.63)	12.4 (±0.60)
14 to 16 years	14.4 (±0.82)	14.6 (±0.87)	14.3 (±0.88)	14.5 (±0.83)

**Table 2:** Inter- and intraobserver reliability for skeletal age assessment.

Modality	Intraclass correlation coefficient: mean (95% CI)		
	Interrater reliability	Intrarater reliability	
	Between raters	Rater 1	Rater 2
Radiographs	0.984 (0.976-0.991)	0.991 (0.982-0.994)	0.989 (0.981-0.995)
MRI	0.976 (0.967-0.992)	0.979 (0.961-0.991)	0.984 (0.971-0.992)

**Table 3:** The mean scores for adequacy of hand positioning as well as image quality for MRI scans and radiographs.

	Radiographs	MRI	*p* value	95% CI
Hand positioning rating (SD)	7.95 (0.68)	5.7 (1.12)	<0.01	(0.52, 1.78)
Image quality rating (SD)	3.87 (0.45)	4.21 (0.24)	0.104	(2.39, 2.93)

## Data Availability

The data used to support the findings of this study are available from the corresponding author upon request.
